# The Risk Factors for Mortality among Septic Trauma Patients: A Retrospective Cohort Study Using the National Trauma Data Bank

**DOI:** 10.1155/2022/6386078

**Published:** 2022-12-30

**Authors:** Nadim Kattouf, Mohamad Assaf, Saadeddine Haidar, Rana Bachir, Mazen El Sayed, Ralph BouChebl

**Affiliations:** Department of Emergency Medicine, American University of Beirut, Beirut, Lebanon

## Abstract

**Introduction:**

In trauma patients, the development of sepsis as a hospital complication is significantly associated with morbidity and mortality. We aimed to assess the risk factors associated with in-hospital mortality among trauma patients who developed sepsis during their hospital stay. *Material and methods*. Using the 2017 National Trauma Data Bank, a retrospective cohort study was conducted to identify adult trauma patients who developed sepsis during their hospital stay. The primary outcome of interest was in-hospital mortality. Multivariate analysis was used to determine the risk factors associated with in-hospital mortality.

**Results:**

1782 trauma patients developed sepsis. 567 patients (31.8%) died during their hospital stay. The following patient factors were associated with higher odds of in-hospital mortality: age (OR = 1.045 95% CI = 1.036–1.054), chronic renal failure (OR = 2.564 95% CI = 1.528–4.301), and liver cirrhosis (OR = 3.699 95% CI = 2.267–6.033). Patients who developed cardiac arrest (OR = 4.994 95% CI = 3.381–7.378), acute kidney injury (OR = 3.808 95% CI = 2.837–5.110), acute respiratory distress syndrome (OR = 1.688 95% CI = 1.197–2.379), and stroke (OR = 1.998 95% CI = 1.075–3.714) during their hospital stay had higher odds of mortality. Higher Glasgow Coma Scale (13–15) at presentation was associated with lower odds of mortality (OR = 0.467 95% CI = 0.328–0.667).

**Conclusion:**

Among trauma patients who developed sepsis, age, chronic renal failure, cirrhosis, the development of cardiac arrest, acute kidney injury, acute respiratory distress syndrome, and stroke in the hospital were associated with in-hospital mortality. These factors can be used to identify patients who are at higher risk of adverse outcomes and implement standardized or protocol-driven methods to improve patient care.

## 1. Introduction

Sepsis and septic shock remains a global public health burden. Sepsis is the most common condition among intensive care unit (ICU) patients [1]. In North America and Europe, it accounts for 10.4% of ICU admissions with an associated 28-day mortality of 36.7% [2]. Trauma, another worldwide public health burden, is a major cause of death for individuals below the age of 44 [3]. In 2014, it resulted in 136053 deaths and was responsible for 29 million Emergency Department (ED) visits in the United States [3]. Multiple factors are associated with worse outcomes in trauma patients who survive initial resuscitation such as sepsis [4, 5]. Loss of tissue integrity and disrupted host defense mechanisms increase infection risk in trauma patients [6–8]. In a study by Eguia et al., six percent (*N* = 320450) of the total trauma population in the United States developed sepsis during their hospital stay [9]. A systematic review showed variability in mortality rates among trauma patients who developed sepsis during their hospital stay; four studies showed a mortality rate of less than seven percent while six others reported a mortality rate of 10% to 23% [10]. Sepsis in trauma patients was associated with an increased overall length of hospital and ICU stay as well as higher rates of single or multiple organ failure [11, 12]. Several risk factors associated with the development of sepsis among trauma patients have been identified. These include injury severity score (ISS), lower Glasgow Coma score (GCS), pre-existing medical conditions, revised trauma score (RTS), age, male gender, number of red blood cell units transfused, and number of operative procedures [11–14].

Studies on the predictors of mortality in trauma patients who develop sepsis during their hospital stay are scarce. The primary aim of the study was to determine the risk factors associated with mortality among trauma patients who develop sepsis during their hospital stay using the National Trauma Data Bank (NTDB). The NTDB collects data on average from one million trauma patients from more than 900 centers yearly and is considered the largest trauma registry in the United States.

## 2. Methods

### 2.1. Study Design

This was a retrospective cohort study conducted by Emergency Medicine faculty members from the American University of Beirut in Lebanon. The 2017 National Trauma Data Bank (NTDB) dataset was used. The NTDB collects data on average from one million trauma patients from more than 900 centers yearly and is considered the largest trauma registry in the United States. This dataset provides insight into prehospital and hospital patient characteristics, hospital complications, outcomes, and trauma-related specifics, such as trauma type and severity [15–17].

All trauma patients admitted to the hospital aged ≥16 who developed sepsis as a hospital complication were included. According to the NTDB, the diagnosis of sepsis must have been documented in the patient's medical record and must have occurred during the patient's initial stay at the hospital. The exclusion criteria were missing age (*N* = 88), ED discharge disposition was not known/not recorded/not applicable (*N* = 97), or transferred to another hospital (*N* = two), and hospital discharge disposition was not known/not recorded (*N* = nine) or underwent interhospital facility transfer (*N* = 633).

### 2.2. Variables of Interest and Outcome

Data regarding patient demographics, comorbidities, trauma characteristics, interventions during hospital stay, hospital complications, and other outcomes (such as ED and hospital disposition and length of hospital stay) were obtained from the database. The primary outcome of interest was in-hospital mortality. The secondary outcomes were ED discharge disposition, length of hospital stay, length of ICU stay, and total mechanical ventilation days.

### 2.3. Statistical Analysis

The statistical package for the social sciences (SPSS, version 24.0; Inc, IBM Corp, Chicago, IL) was adopted to perform all statistical analyses. Continuous variables were summarized by their means and standard deviations, whereas categorical variables were presented through their frequencies and percentages. To compare the patients' demographic and clinical characteristics by outcome (died: yes/no), Pearson's Chi-Square or Fisher's Exact Test and the Mann–Whitney test were used for categorical and continuous variables, respectively. The Shapiro–Wilk test, Kurtosis and Skewness Z-score, and visualization of histograms revealed a violation of the normality distribution of all continuous variables (systolic blood pressure, pulse rate, respiratory rate, pulse oximetry, transfusion blood (4 hours), transfusion blood (24 hours), transfusion platelets (4 hours), transfusion platelets (24 hours), length of stay (days), total ICU length of stay, and total vent days). Therefore, the parametric test “Student's *T* test” was not carried out because none of the continuous variables had a normal distribution and this justified the reason for using the Mann–Whitney test to compare all continuous variables by the outcome (died: yes/no).

A multivariate analysis was conducted to identify the associated factors with patients' mortality. More specifically, a logistic regression model using a stepwise selection method was carried out by controlling for all clinically and statistically significant factors. The variables that were entered into the model were: age (years); sex; race; ethnicity; smoking history; hypertension; diabetes mellitus; chronic renal failure; congestive heart failure; chronic obstructive pulmonary disease (COPD); myocardial infarction (MI); cerebrovascular accident (CVA); peripheral arterial disease (PAD); cirrhosis; disseminated cancer; currently receiving chemotherapy for cancer; bleeding disorder; anticoagulant therapy; functionally dependent health status; steroid use; substance abuse disorder; systolic blood pressure; pulse rate; respiratory rate; pulse oximetry; trauma type; mechanism of injury; nature of injury; body region; signs of life; injury severity score; Glasgow coma scale; blood transfusion (4 hours)—central line-associated bloodstream infection (CLABSI); deep surgical site infection; cardiac arrest with CPR; catheter-associated urinary tract infection (CAUTI); pulmonary embolism; extremity compartment syndrome; unplanned intubation; acute kidney injury; myocardial infarction; organ/space surgical site infection; acute respiratory distress syndrome (ARDS); stroke/CVA; superficial incisional surgical site infection; ventilator-associated pneumonia (VAP). Almost all study variables were included in the multivariate logistic regression except for those having a high percentage of unrecorded data (surgery for hemorrhage control type (72.0%), blood transfusion at 24 hours (72.0%), platelet transfusion at 4 hours (72.3%), and platelet transfusion at 24 hours (72.3%)) and those being as outcomes (such as length of hospital stay, ED discharge disposition, total ICU length of stay, and total ventilation days). The variance inflation factors of all independent variables in the regression model were found to be less than 10, indicating the absence of a multicollinearity problem. The final model was a good fit to the data as indicated by the Hosmer and Lemeshow test (*p*=0.870) and it had a good discrimination between the two categories of outcome (died/survived) as shown by the c-statistic (area under the curve = 0.774; *p* value <0.001; 95% CI: 0.750–0.797). A *p* value of ≤0.05 was used to denote statistical significance.

### 2.4. Missing Data and Outliers

The descriptive analysis showed that the percentage of missing data of all variables was inconsequential because it was less than 5% and therefore it was not handled through multiple imputation procedures. It is worth noting to mention that one of the presented variables “surgery for hemorrhage control type” was not included in the multivariate analysis because it had a very high percentage of unrecorded data (72.0%) that cannot be treated by multiple imputation methods. The Cook's distance of all cases was found to be less than one, revealing that the estimated parameters were not affected by any influential observations.

## 3. Results

The total number of trauma patients included in the database was 997970. A total of 2507 trauma patients who developed sepsis as a hospital complication were identified from the NTDB. After removing the patients who met one of the exclusion criteria, a total of 1782 were included in the data analysis (Figure 1). The average age of all included patients was 56.22 ± 19.64 years. 72.8% were males (*N* = 1298). 31.8% died during their hospital stay (*N* = 567). Nonsurvivors were older than survivors (61.91 ± 18.20 years vs. 53.56 ± 19.73 years, *p* value <0.001). They also had a significantly higher percentage of the following comorbidities: hypertension, diabetes mellitus, chronic renal failure, congestive heart failure, chronic obstructive pulmonary disease, cirrhosis, and malignancy (50.3% vs. 39.2% *p* < 0.001, 25.9% vs. 20.3% *p*=0.008, 9.0% vs. 3.7% *p* < 0.001, 9.9% vs. 6.7% *p*=0.018, 16.9% vs. 12.9% *p*=0.024, 10.2% vs. 3.7% *p* < 0.001, 1.8% vs. 0.7% *p*=0.03, respectively). A higher percentage of nonsurvivors were on anticoagulant therapy (13.8% vs. 10.1%, *p*=0.042) (Table 1).

The percentage of nonsurvivors who presented with a systolic blood pressure less than 90 mmHg was higher compared to survivors (17.2% vs. 12.4%, *p*=0.007). There was no significant difference between both groups with regard to other vital signs at presentation. Trauma type at presentation was significantly different between both groups (*p* < 0.001), with blunt trauma being the most common type of trauma in both groups. The nonsurvivor group had a slightly higher number of blunt trauma patients (85.8% versus 82.5%). The Glasgow Coma Scale at presentation was significantly different between both groups (*p*=0.047), with the nonsurvivors having more patients presenting with aGCS ≤ 8 (22.5% versus 18%). There was no significant difference between both groups with regard to the nature of the injury, body region of injury, injury severity score, and signs of life at presentation (Table 2).

In addition, there was no significant difference in the amount of blood transfusion and platelet transfusion between both groups at 4 and 24 hours after presentation. Similarly, no difference was observed between survivors and nonsurvivors with regard to the type of surgery for hemorrhage control (Table 3).

With regard to hospital complications, the total rates of central line associated blood stream infection, catheter-associated urinary tract infection, and ventilator-associated pneumonia were: 2.2% (*N* = 40), 5.1% (*N* = 91) and 16% (*N* = 286), respectively, (with no statistically significant differences between survivors and nonsurvivors). Nonsurvivors had a higher percentage of cardiac arrest, intubation, acute kidney injury, acute respiratory distress syndrome, and stroke (23.8% vs. 6.2%, *p* < 0.001, 28.7% vs. 22.6% *p*=0.005, 40.4% vs. 17.9% *p* < 0.001, 21.7% vs. 14.3% *p* < 0.001, 5.3% vs. 2.3% *p* < 0.001, respectively). Otherwise, no differences were observed between both groups with regard to other hospital complications (Table 4).

Total hospital length of stay, length of ICU stay, and total ventilation days were significantly higher in the survivor group (33.26 ± 29.38 days vs. 19.59 ± 22.91 days, 20.69 ± 18.39 days vs. 15.28 ± 15.30 days, 17.14 ± 15.77 days vs. 13.89 ± 15.93 days respectively with *p* < 0.001) (Table 5).

In the multivariate analysis, the following variables were found to be associated with in-hospital mortality; age (OR = 1.045, 95% CI = 1.036–1.054, *p* value <0.001), chronic renal failure (OR = 2.564 95% CI = 1.528–4.301 *p* value <0.001) and cirrhosis (OR = 3.699 95% CI = 2.267–6.033, *p* value <0.001). Patients who developed cardiac arrest, acute kidney injury, ARDS, and stroke during their hospital stay had higher odds of mortality (OR = 4.994, 95% CI = 3.381–7.378, *p* value <0.001; OR = 3.808 95% CI = 2.837–5.110, *p* value <0.001; OR = 1.688 95% CI = 1.197–2.379, *p* value =0.003; OR = 1.998 95% CI = 1.075–3.714, *p* value =0.029 respectively). Finally, higher GCS was associated with lower odds of mortality: 13–15 (OR = 0.467, 95% CI = 0.328–0.667, *p* < 0.001) (Table 6).

## 4. Discussion

A total of 1782 trauma patients developed sepsis during their hospital stay and 31.8% (*N* = 567) died throughout. In these patients, age, chronic renal failure, and cirrhosis were found to be associated with in-hospital mortality. Patients who developed cardiac arrest, acute kidney injury, ARDS, and stroke as complications during their hospital stay had higher odds of mortality. Higher GCS was associated with lower odds of mortality.

Various studies reported that age was an independent risk factor associated with in-hospital mortality of sepsis and septic shock, even with adequate early intervention [18–20]. Brakendrige et al. examined the association between age and the innate immune response in a cohort study involving septic trauma and surgery patients. The cohort of aged patients (>55 years old) had worse clinical outcomes and a higher rate of 28-day mortality compared to the young cohort [21]. Increased levels of catabolic biomarkers were reported in the older cohort. The persistence of these biomarkers for up to 28 days indicated a state of immune suppression in older patients with a history of sepsis [21]. In our study, age was also associated with in-hospital mortality in septic trauma patients.

Medical comorbidities have been associated with mortality in sepsis and trauma. The 28-day and 1-year mortality rates of septic shock were higher in patients with CKD compared with non-CKD patients (70% vs. 50%, *p*=0.03, and 82% vs. 64 *p*=0.03, respectively). CKD remained significantly associated with 28-day and 1-year mortality after adjusting for potential confounders [22]. Compared to other comorbidities (including hypertension, history of cancer, diabetes, and liver disease), CKD had the highest hazard ratio for 90-day mortality in a study involving septic caucasian patients (2.25, 95% CI [1.46–3.46]) [23]. Liver cirrhosis, despite advancements in management, remains a risk factor for both trauma and septic shock-related mortality. The mortality rate of cirrhotic patients who develop septic shock was found to range between 60 and 80%, potentially due to the disruption of the innate immune response and excessive stimulation of proinflammatory cytokines [24–27]. Lastly, a study using the National Trauma Data Bank (NTDB) showed a significantly higher mortality rate in patients with cirrhosis (15.8% vs. 8.1%, *p* < 0.0001) and a meta-analysis showed higher odds of mortality for cirrhotic trauma patients compared to noncirrhotic patients (4.52, 95% CI [3.13–6.54]) [28, 29]. In our study, CKD and cirrhosis were associated with in-hospital mortality in septic trauma patients.

The results of this study have shown that septic trauma patients with higher GCS scores had lower odds of in-hospital mortality (OR = 0.467, 95% CI = 0.328–0.667, *p* < 0.001 for GCS = 13–15 compared to ≤8). Historically, The Glasgow Coma Score has been found to be associated with increased mortality in trauma patients. Sewalt et al. identified 154476 patients between 2013 and 2016 from the Trauma Audit and Research Network. They found that the GCS score was among the three most important predictors of in-hospital mortality [30]. It is possible that lower GCS patients are perceived as higher-risk patients who would require more prompt and aggressive care, as well as better monitoring and followup in the hospital.

Septic trauma patients who had a history of cardiac arrest or stroke during their hospital stay were found to have higher mortality. Postsepsis, MI, or stroke was independently associated with increased 180-day (HR = 2.16, 95% CI 1.69–2.76) and 365-day (HR = 1.90, 95% CI 1.54–2.32) mortality [31]. In addition, traumatic cardiac arrest is associated with poor outcomes; studies have reported overall survival rates of 2.6% and 5.6% [32, 33]. In another study, patients who developed stroke after a traumatic brain injury had higher mortality rates than those who only sustained a TBI (10.2% vs. 3.2%, *p* < 0.0001) with an adjusted relative risk of death (RR) of 1.46 (95% CI = 1.15–1.84) [34]. Similarly in our study, the development of cardiac arrest or stroke among septic trauma patients during hospital stay was associated with increased mortality.

In critically ill patients, acute kidney injury (AKI) is a common complication and is associated with increased mortality [35]. Sepsis is one of the major contributors to the development of AKI in critically ill patients [36]. In a study of 5680 septic and septic shock patients, 57.7% developed AKI. The AKI group had a higher mortality rate (16.4% vs. 2.9%) and increased AKI severity was associated with increased mortality [37]. Trauma is also a major contributor to the development of AKI [38, 39]. Out of 413 trauma patients admitted to the ICU of a level 1 trauma center, 24.9% developed AKI during the first week. AKI was associated with an increase in 30-day (17.5% vs. 5.8%) and 1 year mortality (26.2% vs. 7.1%) [38]. In a meta-analysis of 25,182 trauma patients admitted to the ICU, the incidence of AKI was 24% [39]. Trauma patients who developed AKI had a significantly higher length of ICU stay and risk of death (RR = 3.4) [39]. Similarly, in our study, septic trauma patients who developed AKI during their hospital stay had higher odds of in-hospital mortality.

Finally, Sepsis is the most common cause of ARDS [40]. In a study by Mikkelsen et al., the incidence of ARDS among septic patients was 6.2%. Patients who developed ARDS had higher rates of in-hospital mortality (60% vs. 14%) [41]. Traumatic injury represents the third most common cause of ARDS [42]. In a study using the 2010–2014 national Trauma quality improvement dataset, the incidence of ARDS went from 3% to 1.1%, but associated mortality increased (18% to 21%, *p* < 0.001) [43]. Severe traumatic brain injury patients were found to have an incidence of 20–25% for ARDS. ARDS in those patients was associated with increased mortality [44]. Similarly, in our study, septic trauma patients who developed ARDS during their hospital stay had higher odds of in-hospital mortality.

Finally, older age, CKD, and cirrhosis put trauma patients who develop sepsis in a higher risk category. These patients may benefit from more frequent and careful monitoring and management. Similarly, septic trauma patients who develop AKI, cardiac arrest, stroke, or ARDS have a poor prognosis, and aggressive management to prevent these conditions should occur in the ICU setting.

## 5. Limitations

One of the limitations of this study is its retrospective nature. To obtain our sample, we used ICD-10 CM for trauma and sepsis. There can be variations in coding from one hospital to another. This can affect the selection of the sample by not including all eligible septic trauma patients. Patients with a missing disposition from the ED were excluded; this can lead to selection bias. Our study included patients with a diagnosis of sepsis on their medical record. Sepsis-3 criteria were not used thus some patients with sepsis may have not been included. There were some potential confounders that we would have liked to adjust for but were missing from the database, such as laboratory parameters, imaging results, etiology of sepsis, and sepsis severity scores. In addition, the database only includes hospitals located in the United States, which can limit the generalizability of this study to other populations. However, this database consists of the largest trauma registry in the United States, making the results of this study generalizable to the United States health system. There might be differences in the data quality collected from the different hospitals in the NTDB. Despite these limitations, the data is under continuous monitoring and reviewing in order to maintain its high quality.

## 6. Conclusion

This retrospective study was conducted using data obtained from the NTDB. We aimed to identify predictors of in-hospital mortality among trauma patients who develop sepsis as a hospital complication. Older Age, CKD, liver cirrhosis, and the development of cardiac arrest, stroke, AKI, and ARDS were associated with increased in-hospital mortality. A higher GCS score was associated with decreased odds of in-hospital mortality.

## Figures and Tables

**Figure 1:** Flow diagram showing the inclusion and exclusion criteria of this study in addition to the total number of patients included in the analysis. ^*∗*^Note: There are overlaps among the categories of the excluded variables. More specifically, some patients who had interhospital facility transfer had an ED disposition as one of the excluded categories. Also, some patients whose age was not recorded or were 15 years or younger were transferred or had an ED disposition as one of the excluded categories. These overlaps explain why the final number on which the data analysis was conducted cannot be calculated just by subtracting the number of excluded patients from the selected sample. *∗*Note: There are overlaps among the categories of the excluded variables. More specifically, some patients who had interhospital facility transfer had an ED disposition as one of the excluded categories. Also, some patients whose age was not recorded or were 15 years or younger were transferred or had an ED disposition as one of the excluded categories. These overlaps explain why the final number on which the data analysis was conducted cannot be calculated just by subtracting the number of excluded patients from the selected sample.

**Table 1:** Table showing the baseline characteristics of the trauma patients who developed sepsis during their hospital stay.

	Total	Died		*p* value
	*N* = 1782	No (*N* = 1215)	Yes (*N* = 567)	
Age (years)				
16–25	160 (9.0%)	130 (10.7%)	30 (5.3%)	<0.001
26–35	187 (10.5%)	151 (12.4%)	36 (6.3%)	
36–45	187 (10.5%)	146 (12.0%)	41 (7.2%)	
46–55	248 (13.9%)	187 (15.4%)	61 (10.8%)	
56–65	363 (20.4%)	224 (18.4%)	139 (24.5%)	
≥66	637 (35.7%)	377 (31.0%)	260 (45.9%)	
Age	56.22 ± 19.64	53.56 ± 19.73	61.91 ± 18.20	<0.001
Sex				
Male	1298 (72.8%)	895 (73.7%)	403 (71.1%)	0.242
Female	483 (27.1%)	319 (26.3%)	164 (28.9%)	
Not known/Not recorded	1 (0.1%)			
Race				
Black	312 (17.5%)	220 (18.5%)	92 (16.6%)	0.154
White	1231 (69.1%)	823 (69.2%)	408 (73.5%)	
Other race^1^	202 (11.3%)	147 (12.4%)	55 (9.9%)	
Not known/Not recorded	37 (2.1%)			
Ethnicity				
Hispanic or latino	192 (10.8%)	132 (11.5%)	60 (10.9%)	0.752
Not hispanic or latino	1507 (84.6%)	1019 (88.5%)	488 (89.1%)	
Not known/Not recorded	83 (4.7%)			
Current smoker	405 (22.7%)	297 (24.4%)	108 (19.0%)	0.011
Hypertension	761 (42.7%)	476 (39.2%)	285 (50.3%)	<0.001
Diabetes mellitus	394 (22.1%)	247 (20.3%)	147 (25.9%)	0.008
Chronic renal failure	96 (5.4%)	45 (3.7%)	51 (9.0%)	<0.001
Congestive heart failure	137 (7.7%)	81 (6.7%)	56 (9.9%)	0.018
Chronic obstructive pulmonary disease (COPD)	253 (14.2%)	157 (12.9%)	96 (16.9%)	0.024
Myocardial infarction (MI)	28 (1.6%)	16 (1.3%)	12 (2.1%)	0.206
Cerebrovascular accident (CVA)	75 (4.2%)	51 (4.2%)	24 (4.2%)	0.972
Peripheral arterial disease (PAD)	24 (1.3%)	15 (1.2%)	9 (1.6%)	0.547
Cirrhosis	103 (5.8%)	45 (3.7%)	58 (10.2%)	<0.001
Disseminated cancer	18 (1.0%)	8 (0.7%)	10 (1.8%)	0.030
Currently receiving chemotherapy for cancer	16 (0.9%)	10 (0.8%)	6 (1.1%)	0.624
Bleeding disorder	59 (3.3%)	36 (3.0%)	23 (4.1%)	0.230
Anticoagulant therapy	205 (11.5%)	127 (10.5%)	78 (13.8%)	0.042
Functionally dependent health status	198 (11.1%)	123 (10.1%)	75 (13.2%)	0.052
Steroid use	37 (2.1%)	24 (2.0%)	13 (2.3%)	0.662
Substance abuse disorder	192 (10.8%)	142 (11.7%)	50 (8.8%)	0.069

**Table 2:** Table showing the baseline vital signs, trauma characteristics, and state of presentation of trauma patients who developed sepsis during their hospital stay.

	Total	Died		*p* value
	*N* = 1782	No (*N* = 1215)	Yes (*N* = 567)	
Systolic blood pressure				
≤90	242 (13.6%)	147 (12.4%)	95 (17.2%)	0.007
≥91	1497 (84.0%)	1040 (87.6%)	457 (82.8%)	
Not known/Not recorded	43 (2.4%)			
Systolic blood pressure (mmHg)	128.39 ± 35.522	129.05 ± 34.425	126.98 ± 37.769	0.262^*∗∗*^
Pulse rate (Beats/minute)	97.46 ± 25.52	98.27 ± 25.30	95.70 ± 25.90	0.093^*∗∗*^
Respiratory rate (Breaths/minute)	20.31 ± 6.58	20.25 ± 6.55	20.45 ± 6.63	0.960^*∗∗*^
Pulse oximetry (% saturation)	95.48 ± 7.82	95.46 ± 8.13	95.52 ± 7.09	0.659^*∗∗*^
Trauma type				
Blunt	1479 (83.0%)	995 (82.5%)	484 (85.8%)	<0.001
Penetrating	222 (12.5%)	173 (14.3%)	49 (8.7%)	
Burn	69 (3.9%)	38 (3.2%)	31 (5.5%)	
Not known/Not recorded	12 (0.7%)			
Mechanism of injury				
Fall	693 (38.9%)	453 (37.6%)	240 (43.1%)	0.011
Firearm	182 (10.2%)	142 (11.8%)	40 (7.2%)	
MVT	636 (35.7%)	433 (36.0%)	203 (36.4%)	
Other^2^	250 (14.0%)	176 (14.6%)	74 (13.3%)	
Not known/Not recorded	21 (1.2%)			
Nature of injury				
Fracture	691 (38.8%)	478 (39.6%)	213 (37.8%)	0.922
Internal organ injury	695 (39.0%)	468 (38.8%)	227 (40.2%)	
Open wound	129 (7.2%)	90 (7.5%)	39 (6.9%)	
Superficial and contusion	102 (5.7%)	68 (5.6%)	34 (6.0%)	
Other^3^	154 (8.6%)	103 (8.5%)	51 (9.0%)	
Not known/Not recorded	11 (0.6%)			
Body region				
Extremities	428 (24.0%)	291 (24.1%)	137 (24.3%)	0.424
Head and neck	551 (30.9%)	367 (30.4%)	184 (32.6%)	
Spine and back	173 (9.7%)	119 (9.9%)	54 (9.6%)	
Torso	576 (32.3%)	405 (33.6%)	171 (30.3%)	
Unclassifiable by body region & unspecified	43 (2.4%)	25 (2.1%)	18 (3.2%)	
Not known/Not recorded	11 (0.6%)			
Signs of life				
Arrived with no signs of life	9 (0.5%)	4 (0.3%)	5 (0.9%)	0.154*∗*
Arrived with signs of life	1773 (99.5%)	1211 (99.7%)	562 (99.1%)	
ISS				
≤15	759 (42.6%)	531 (43.7%)	228 (40.4%)	0.179
≥16	1020 (57.2%)	683 (56.3%)	337 (59.6%)	
Not known/Not recorded	3 (0.2%)			
GCS				
Severe ≤8	331 (18.6%)	207 (18.0%)	124 (22.5%)	0.047
Moderate 9–12	126 (7.1%)	81 (7.0%)	45 (8.2%)	
Mild 13–15	1244 (69.8%)	862 (75.0%)	382 (69.3%)	
Not known/Not recorded	81 (4.5%)			

^3^Other nature of injury includes: Amputation & Blood vessel & Burns and corrosions & Crushing & Dislocation & Other effects of external causes & Other specified injury & Toxic effects & Unspecified injury. ^*∗*^ Indicates that Fisher's exact was used to calculate the *p* value. ^*∗∗*^ Indicates that the Mann–Whitney test was used to calculate the *p* value.

**Table 3:** Table showing the therapeutic interventions undergone by the trauma patients who developed sepsis during this hospital stay.

	Total	Died		*p* value
	*N* = 1782	No (*N* = 1215)	Yes (*N* = 567)	
Transfusion blood (4 Hours) (mL)	423.96 ± 1297.02	452.02 ± 1375.48	368.67 ± 1128.43	0.735^*∗∗*^
Transfusion blood (24 Hours) (mL)	659.47 ± 2202.30	653.85 ± 2163.05	670.54 ± 2284.21	0.992^*∗∗*^
Transfusion platelets (4 Hours) (mL)	76.61 ± 201.50	79.79 ± 210.92	70.71 ± 183.76	0.439^*∗∗*^
Transfusion platelets (24 Hours) (mL)	116.83 ± 340.84	106.22 ± 304.89	136.32 ± 399.44	0.190^*∗∗*^
Surgery for hemorrhage control type				
None	176 (9.9%)	117 (35.3%)	59 (35.1%)	0.557*∗*
Laparotomy	252 (14.1%)	169 (51.1%)	83 (49.4%)	
Thoracotomy	20 (1.1%)	13 (3.9%)	7 (4.2%)	
Sternotomy	3 (0.2%)	1 (0.3%)	2 (1.2%)	
Extremity	22 (1.2%)	17 (5.1%)	5 (3.0%)	
Neck	2 (0.1%)	1 (0.3%)	1 (0.6%)	
Mangled extremity/traumatic amputation	11 (0.6%)	7 (2.1%)	4 (2.4%)	
Other skin/soft tissue	13 (0.7%)	6 (1.8%)	7 (4.2%)	
Not known/Not recorded	1283 (72.0%)			

^*∗*^ Indicates that Fisher's exact was used to calculate the *p* value. ^*∗∗*^ Indicates that the Mann–Whitney test was used to calculate the *p* value.

**Table 4:** Table showing the hospital complications experienced by the trauma patients who developed sepsis during their hospital stay.

	Total	Died		*p* value
	*N* = 1782	No (*N* = 1215)	Yes (*N* = 567)	
Central line-associated bloodstream infection (CLABSI)	40 (2.2%)	27 (2.2%)	13 (2.3%)	0.925
Deep surgical site infection	65 (3.6%)	49 (4.0%)	16 (2.8%)	0.204
Cardiac arrest with CPR	210 (11.8%)	75 (6.2%)	135 (23.8%)	<0.001
Catheter-associated urinary tract infection (CAUTI)	91 (5.1%)	63 (5.2%)	28 (4.9%)	0.825
Pulmonary embolism	66 (3.7%)	51 (4.2%)	15 (2.6%)	0.106
Extremity compartment syndrome	19 (1.1%)	14 (1.2%)	5 (0.9%)	0.605
Unplanned intubation	438 (24.6%)	275 (22.6%)	163 (28.7%)	0.005
Acute kidney injury	446 (25.0%)	217 (17.9%)	229 (40.4%)	<0.001
Myocardial infarction	63 (3.5%)	36 (3.0%)	27 (4.8%)	0.055
Organ/Space surgical site infection	57(3.2%)	42 (3.5%)	15 (2.6%)	0.365
Acute respiratory distress syndrome (ARDS)	297 (16.7%)	174 (14.3%)	123 (21.7%)	<0.001
Stroke/CVA	58 (3.3%)	28 (2.3%)	30 (5.3%)	0.001
Superficial incisional surgical site infection	36 (2.0%)	31 (2.6%)	5 (0.9%)	0.020
Ventilator-associated pneumonia (VAP)	286 (16.0%)	184 (15.1%)	102 (18.0%)	0.127

**Table 5:** Table showing the hospital outcomes of the trauma patients who developed sepsis during their hospital stay.

	Total	Died		*p* value
	*N* = 1782	No (*N* = 1215)	Yes (*N* = 567)	
ED discharge disposition				0.066*∗*
Floor bed (general admission, nonspecialty unit bed)	345 (19.4%)	251 (20.7%)	94 (16.6%)	
Observation unit (unit that provides <24 hour stays)	18 (1.0%)	11 (0.9%)	7 (1.2%)	
Telemetry/step-down unit (less acuity than ICU)	106 (5.9%)	65 (5.3%)	41 (7.2%)	
Operating room	491 (27.6%)	345 (28.4%)	146 (25.7%)	
Intensive care unit (ICU)	819 (46.0%)	540 (44.4%)	279 (49.2%)	
Home without services	3 (0.2%)	3 (0.2%)	0 (0%)	
Length of stay (days)	29.13 ± 28.28	33.26 ± 29.38	19.59 ± 22.91	<0.001^*∗∗*^
Total ICU length of stay (days)	18.87 ± 17.59	20.69 ± 18.39	15.28 ± 15.30	<0.001^*∗∗*^
Total vent days	15.95 ± 15.89	17.14 ± 15.77	13.89 ± 15.93	<0.001^*∗∗*^

^*∗*^ Indicates that Fisher's exact was used to calculate the *p* value. ^*∗∗*^ Indicates that the Mann–Whitney test was used to calculate the *p* value.

**Table 6:** Table showing the risk factors for mortality in trauma patients who developed sepsis during their hospital stay.

	Adjusted odds ratio^*∗*^	95% CI	*p* value
Age (years)	1.045	1.036–1.054	<0.001
GCS (Severe ≤ 8)			
Moderate 9–12	0.683	0.392–1.188	0.177
Mild 13–15	0.467	0.328–0.667	<0.001

*Comorbidities*			
Chronic renal failure (No)			
Yes	2.564	1.528–4.301	<0.001
Cirrhosis (No)			
Yes	3.699	2.267–6.033	<0.001

*Hospital complications*			
Cardiac arrest with CPR (No)			
Yes	4.994	3.381–7.378	<0.001
Acute kidney injury (No)			
Yes	3.808	2.837–5.110	<0.001
Acute respiratory distress syndrome (ARDS) (No)			
Yes	1.688	1.197–2.379	0.003
Stroke/CVA (No)			
Yes	1.998	1.075–3.714	0.029

^*∗*^Variables entered into the model: Age (years)—Sex—Race—Ethnicity—Comorbidities [current smoker; hypertension; diabetes mellitus; chronic renal failure; congestive heart failure; chronic obstructive pulmonary disease (COPD); myocardial infarction (MI); cerebrovascular accident (CVA); peripheral arterial disease (PAD); cirrhosis; disseminated cancer; currently receiving chemotherapy for cancer; bleeding disorder; anticoagulant therapy; functionally dependent health status; steroid use; substance abuse disorder]—sbp—pulse rate—respiratory rate—pulse oximetry—trauma type—mechanism of injury—nature of injury—body region—signs of life—iss—gcs—transfusion blood (4 hours)—hospital complications [Central line-associated bloodstream infection (CLABSI); deep surgical site infection; cardiac arrest with cpr; catheter-associated urinary tract infection (CAUTI); pulmonary embolism; extremity compartment syndrome; unplanned intubation; acute kidney injury; myocardial infarction; organ/space surgical site infection; acute respiratory distress syndrome (ARDS); stroke/CVA; superficial incisional surgical site infection; ventilator-associated pneumonia (VAP)].

## Data Availability

The datasets used and/or analyzed during the current study are available from the corresponding author upon reasonable request.
